# A Novel Robotic Exoskeleton for Finger Rehabilitation: Kinematics Analysis

**DOI:** 10.1155/2022/1751460

**Published:** 2022-10-14

**Authors:** Yong Dai, Junhong Ji, Guocai Yang, Yu Yang

**Affiliations:** ^1^School of Mechatronics Engineering, Harbin Institute of Technology, Harbin 150001, China; ^2^State Key Laboratory of Robotics and Systems, Harbin Institute of Technology, Harbin 150001, China

## Abstract

A novel robotic exoskeleton for fingers rehabilitation is developed, which is driven by linear motors through Bowden cables. For each finger, in addition to three links acting as phalanxes, two more links acting as knuckles are also implemented. Links are connected through passive joints, by which translational and rotary movements can be realized simultaneously. Either flexion or extension motion is accomplished by one cable of adequate stiffness. This exoskeleton possesses good adaptability to finger length of different subjects and length variations during movement. The exoskeleton's kinematics model is built by the statistics method, and piecewise polynomial functions (PPF) are chosen to describe the relationship between motor displacement and joint variables. Finally, the relationship between motor displacement and the finger's total bending angle is obtained, which can be used for rehabilitation trajectory planning. Experimental results show that this exoskeleton achieves nearly the maximum finger bending angle of a healthy adult person, with the maximum driving force of 68.6 N.

## 1. Introduction

The human hand is one of the most sophisticated human body parts performing many activities of daily living, so the life quality of patients suffering impairments in hand function is badly affected. Due to the huge amount of patients after stroke or spine injury, the demand for rehabilitation therapy to regain normal hand strength and capabilities is huge [1, 2]. In past, such a rehabilitation process was executed manually by physiotherapists. As technology improves, robot-aided hand rehabilitation or assisting devices have conveyed a lot of interest and have been proven to be good as or even better than conventional therapy because of providing high-intensity and repetitive therapy [3, 4]. With help of robots, patients could practice more easily at their own will and handle functional daily living tasks at ease.

Some prototypes or even commercial products have been developed, which can be categorized into three major types, that is, based on end-effector, exoskeleton, or just a glove, respectively. With the former one, it is usually impossible to control each joint involved in the motion [5], so most current systems are in the form of exoskeleton. The exoskeleton is generally a mechanism that can be placed around a part of the human body to mechanically guide or actuate it without impeding the joint's natural motion [5]. Exoskeletons can be categorized into different types depending on various criteria, comprehensive categorization with respect to exoskeleton is provided in [6]. Major criteria include actuator type, intention sensing method, purpose, and power transmission methods. According to the actuator type, an exoskeleton can be driven by electric motors, pneumatic pistons, pneumatic air chambers, pneumatic artificial rubber muscles (PARMs), series elastic actuators (SEA), shape memory alloy (SMA), and hydraulics for active systems. According to the power transmission method, structures can be driven directly by actuators or with the aid of linkage, belt, cable-driven tendon, or cable with linkages together [4]. Obviously, there are much more combinations than the above-listed categories, for instance, the torque exerted via linkage can be from either an electric motor or SMA.

Linkage is the most conventional way consisting an exoskeleton [7–10]. The essential weakness is that the structure is bulky, especially on the dorsal side. To adapt to various finger sizes, a linkage exoskeleton was developed, whose mechanism's active joint axes do not have to coincide with the finger joint axes of human hands [11], with the cost of an extreme bulky mechanical structure.

To modulate mechanic length to adapt finger flexion/extension, a sliding mechanism is adopted. A three-layered sliding spring mechanism is developed to realize large deformation [5]. For each joint, when the inner spring bends, the center and outer springs bend and actively and passively slide, respectively, forming a circular sector. This structure is quite complicated and the stiffness of springs should be chosen carefully. Another common way to adapt different lengths of patients' fingers is implementing passive prismatic joints in addition to active rotary joints [2, 12–15]. Such structure is also helpful to align finger joints and rotary centers.

A slider-crank-like mechanism is proposed to transmit driving torque onto the metacarpophalangeal (MCP) joint, while proximal interphalangeal (PIP) and distal interphalangeal (DIP) are driven by the Bowden cable. Shell-like structures are fastened on fingers and palms by Velco straps. Two passive translational joints are involved to adapt the finger length of different subjects after manually adjusting such joints are blocked by the screw [2]. A similar linkage structure can be also actuated by SMA instead of electric motors [16].

The principle of remote center of motion (RCM) is another way to fit the mechanical rotation center to human joints. This can be realized by multiparallelogram linkages [17], arc-shaped sliders [18], N-shaped linkages [19], or even more complicated structures consisting of 2 four-bar linkages and 3 five-bar linkages [20]. The common drawback is still that the mechanical structure is bulky and complicated.

Cable is an attractive way of mimicking the tendon's physiological function, while just unidirectional torque can be exerted by one cable [21]. To exert bidirectional torque on one finger, either two independent cables [22] or a pulley is implemented [23]. To replace the pulley, a U-shaped tube can also be implemented to guide wires as tendons for extension and flexion [24], while extension wires are attached to linear springs to generate extension force. The Bowden cable–based series elastic actuation (SEA) is developed allowing bidirectional torque control [1]. Although low reflected inertia is realized to offer minimal resistance to finger motion, the dimension is still big. Sliding joints are implemented as the interface between finger phalanx and exoskeleton links, which can be quickly adjusted, that is, it is still needed adjusting for the individual subject. An exoskeleton driven by cable can cover more than 70% of a healthy hand workspace, and it can achieve forces at the fingertips sufficient for activities of daily living [25]. HX-*β*, an index finger-thumb exoskeleton is driven by series-elastic actuators via cables, realized robot-user joint alignment, and flexible actuation for users of various hand sizes [26]. In a prototype named “RELab tenoexo,” sleek mechanisms are designed, which can generate the four most frequently used grasp motions [27]. A SEA-based prototype is developed which incorporates five passive and two actively actuated joints and provides active control of MCP and PIP joints. But the structure is still bulky; therefore, only the part for index finger is realized [28].

To obtain force feedback in an exoskeleton, whose original purpose is for virtual reality, two cables are implemented, one cable for driving and another one for force feedback [29].

Pneumatic actuators are widespread because of advantages such as high weight–power ratio, compressibility, low heat generation, and clean energy, while a primary drawback is that only unidirectional force/torque can be exerted. A McKibben type pneumatic artificial muscle (PAM) is implemented for actuation [30], to overcome the unidirectional drawback, it is combined with a constant force spring. PARMs are also adopted in grip amplified glove, which achieves power-assist grasping motion [31], but are unhelpful for flexor hypertonia.

Since many patients have flexor hypertonia and finger extensor weakness, a passive exoskeleton, which can exert only unidirectional extension torque, is also developed. Series of elastic cords [32], passive leaf springs, and elastic tension cords [33] are adopted against excessive involuntary flexion torques due to impairments. To apply such a device, offset force should be manually adjusted in advance.

Bio-signals are a way to detect the users' intentions by measuring electrical muscle activity in the forearm or motor functions in the brain. Surface electromyography (SEMG) can be used as a sensor to control the exoskeleton or observe and get feedback from the progress of training. SEMG signals combined with kinematic information from exoskeleton's encoders can be introduced to a torque-controlled hand exoskeleton [34].

The glove is an intuitive and compact embodiment of the wearable device. A polymer-based tendon-driven wearable robotic hand permits adjustment to different hand sizes and ventilation [35].

The soft robot is also an attractive way. A prototype made of molded elastomeric bladders with anisotropic fiber reinforcement was built, which can produce specific bending, twisting, and extending trajectories upon fluid pressurization [36, 37]. It can be quickly custom-designed to fit the anatomy of individual users, that is, soft actuators were mechanically programmed to match and support the range of motion of individual fingers. Given the condition that soft devices tend to lack well-understood models and traditional rigid devices are always with excessive stiffness, a hybrid soft-rigid exoskeleton (HSRexo) is presented, adopting the simplified three-layered sliding spring (sTLSS) mechanism that combines the intrinsic compliance and comprehensible kinematics [38].

As a common difficulty is that, without correct alignment, the exoskeleton will feel uncomfortable in use, or even unusable [39], a feasible solution is proposed to automatically align exoskeleton axes to human anatomical axes by decoupling joint rotations from translations [40].

In most existing exoskeletons, the adaptability to different patients' fingers is deficient. For some devices, the finger's total bending angle is still inadequate, besides the wearing procedure is a burdensome task, which may last for 30 minutes.

To summarize, there are still several challenges to overcome, that is, an ideal exoskeleton should be:

- compact in size to minimize the interference between the thumb and fingers
- easy to wear
- adaptable to different patients' finger lengths
- adjustable in length during flexion/extension to minimize the slippage between the finger phalanx and exoskeleton links

To overcome such drawbacks, a novel exoskeleton is developed, for which each finger is driven by an individual linear motor through a Bowden cable. For each finger, two more links are implemented as knuckles. Links are connected by passive joints; therefore, rotational and translational movements can be realized simultaneously. For human knuckles, wrinkles play a vital role to modulate skin tension during movement. In this exoskeleton, knuckle links will lead to adaptability to different subject finger lengths and motion diversity. Compared to the combination of active rotary joint and passive prismatic joint, the designed passive joint can realize rotary and translational movements simultaneously. As a consequence, the mechanical structure is more compact. For this structure, a finger's configuration is described by eight variables. With a cable possessing adequate stiffness, finger flexion/extension is achieved by cable push/pull action. Since there is only one active input, this exoskeleton performs as a typical single input–multiple output system. Theoretically, given a determinate motor displacement, there are infinite possible finger configurations. To build a feasible direct kinematics model for control purposes, the statistic method is implemented. As a consequence, the piecewise polynomial function is adopted to describe the mapping from motor displacement to those variables.

The rest of this article is organized as follows. The hardware structure is introduced in the next section, followed by the kinematics model and parameter estimation process; afterward, experimental results are provided, and finally, the conclusion is given.

## 2. Hardware Structure

Based on an investigation of patients' demand and feeling, two issues are recognized as important. First, slippage between the finger and exoskeleton during movement should be minimized. Second, the exoskeleton should adopt different patients' finger lengths and length variations during movement. Motivated by those issues, a novel exoskeleton is designed, which consists of a palm platform and five finger assemblies. Then, a textile glove will be adhered to the exoskeleton's bottom side by glue. The exoskeleton mechanism is demonstrated in Figure 1.

### 2.1. Mechanical Parts

The mechanical structure for one finger is shown in Figure 2, which is consisted of one fixed link (no. 0) and five moveable links. Imitating a human being's hand, moveable links are categorized as phalanxes (no. 1, 3, 5) and knuckles (no. 2, 4). When the finger is totally extended, knuckles locate completely inside adjacent phalanxes. On links no. 1 and 3, one and two slots are milled, respectively. Hinges fixed on adjacent links can move freely inside those slots, either rotating or translating. Due to such structure, the exoskeleton can passively adapt to the patient finger's geometrical variation, both flexing angle and length.

A path for the Bowden cable is formed by tunnels inside links no. 0, 2, and 4 (area without section lines in Figure 2(b)). One end of the cable is connected to a linear motor (see Figure 3), and another end is fixed inside the fingertip. When the cable is pushed or pulled by the motor, the finger will be flexed or extended.

To realize both flexion and extension action by one cable, certain cable stiffness is compulsory. This is ensured by two aspects: on the one hand, a cable with a diameter of 2.5 mm is chosen among cables with different diameters. More importantly, almost the complete cable is constrained by surrounding structures: metal sleeve, rigid plastic tube (see Figure 3), and tunnels mentioned above. The linear motor's shaft is connected to a rod, which moves inside a sleeve. Along the complete cable, the maximum lateral tolerance is about 4 mm, which takes place inside the tunnel. As a consequence, adequate stiffness of the cable is achieved to exert bidirectional torques. A preliminary experiment shows that given the maximum motor displacement of 80 mm, the maximum displacement error due to cable bending is less than 2 mm.

### 2.2. Electronic Part

Each finger is driven by an individual linear motor, whose displacement is directly controlled, given maximum velocity and acceleration restrictions. During the rehabilitation process, fingers usually move slowly, and the dynamic characteristics of both finger and mechanism are not considered; in other words, it is adequate to control the motor in a displacement way, if the motor's output torque is sufficient.

A dyadic SCN5 series linear motor is adopted, whose driver communicates with a host computer via RS-485 bus according to the dyadic Termi-BUS protocol (see Figure 4). To realize closed-loop control, instructions are sent to motor drivers in turn through COM1 port, while the motor position and working status are read through COM2 port.

To monitor force through the Bowden cable, a ZNLBM-VII force sensor (with a resolution of 0.06 N in the range of 0–200 N) is installed between the motor shaft and the connecting rod (see Figure 3). Compared to the solution adopting another cable for force feedback [22], this method is more compact and reliable, since force is measured directly on the drive cable. At the present stage, only motor displacement control is implemented. Cable force will be implemented to realize impedance control in the next step.

## 3. Kinematics Model

### 3.1. Definition of Coordinate Frames

Taking the forefinger as an instance, for each link, a local coordinate frame, involving *x* and *y* axes, is defined (see Figure 2(a)). At initial configuration, that is, while the finger is totally extended, all frames' *x* and *y* axes are toward right and up, respectively. Origins of frames no. 0 and 1 are located at the same position, that is, the hinge connecting them. Origins of frames no. 2, 4, and 5 are located at corresponding proximal hinges. A little attention should be paid to frame no. 3, because there is no hinge fixed on link no. 3. The origin locates at the most proximal position for the distal hinge on link no. 2. Relative orientation and displacement between adjacent frames can be described by two quantities *θ*_*i*_ and *d*_*i*_ (see Table 1). Angle *θ*_*i*_ represents the angle from the axis *x*_*i*_ to axis *x*_*i*−1_, counterclockwise. *d*_*i*_ is the displacement of the origin *o*_*i*+1_ along the axis *x*_*i*_. As instance, *θ*_1_ and *d*_1_ are depicted in Figure 5. Note, *d*_2_ and *d*_5_ are constants, that is, distances between two hinges on link no. 2 and 4, respectively.

According to the definition of *θ*_*i*_ and *d*_*i*_, the homogeneous transformation matrices between consequent link coordinate frames are given as:

(1) $$\begin{array}{c} T_{1}^{0}=\left[\begin{array}{ccc} \cos\theta_{1} & -\sin\theta_{1} & 0\\ \sin\theta_{1} & \cos\theta_{1} & 0\\ 0 & 0 & 1 \end{array}\right], \end{array}$$

(2) $$\begin{array}{c} T_{2}^{1}=\left[\begin{array}{ccc} \cos\theta_{2} & -\sin\theta_{2} & d_{1}\\ \sin\theta_{2} & \cos\theta_{2} & 0\\ 0 & 0 & 1 \end{array}\right], \end{array}$$

(3) $$\begin{array}{c} T_{3}^{2}=\left[\begin{array}{ccc} \cos\theta_{3} & -\sin\theta_{3} & d_{2}+d_{3}\cos\theta_{3}\\ \sin\theta_{3} & \cos\theta_{3} & d_{3}\sin\theta_{3}\\ 0 & 0 & 1 \end{array}\right], \end{array}$$

(4) $$\begin{array}{c} T_{4}^{3}=\left[\begin{array}{ccc} \cos\theta_{4} & -\sin\theta_{4} & d_{4}\\ \sin\theta_{4} & \cos\theta_{4} & 0\\ 0 & 0 & 1 \end{array}\right], \end{array}$$

(5) $$\begin{array}{c} T_{5}^{4}=\left[\begin{array}{ccc} \cos\theta_{5} & -\sin\theta_{5} & d_{5}\\ \sin\theta_{5} & \cos\theta_{5} & 0\\ 0 & 0 & 1 \end{array}\right]. \end{array}$$

### 3.2. Direct Kinematics Model

Taking the motor's displacement as input, as mentioned above, there are eight output variables, so the finger mechanism acts as a typical single-input multi-outputs system. Theoretically, there are infinite solutions, affected by many factors, for example, the patient finger's dimension, muscular tension, friction, etc. It is extremely difficult to find an analytical solution. Preliminary experiments show that, cooperated with the same subject, the exoskeleton motion's repeatability is quite good, which inspires us implementing statistic characteristics as the direct kinematics model.

To build the statistic kinematics model, images are acquisitioned. Given the linear motor's displacements as inputs, corresponding image series are taken. Five markers have been attached to the exoskeleton, which are denoted by marker no. 1–5 (see Figure 6). Pixel locations corresponding to centers of hinges and markers are read by image editing software. As mentioned early, *d*_2_ is a constant, that is, the distance between two hinges on link no. 2. Knowing the ratio between the pixel distance and real length, another translational displacement can be calculated, for example, *d*_1_ and *d*_4_. Again, a little more attention is paid to *d*_3_, because there is no fixing point on link no. 3 corresponding to the origin of the link coordinate frame no. 3. So, the origin's position is determined with help of markers no. 1 and 2, since marker no. 2 is placed at the midpoint of the line segment connecting marker no. 1 and the origin of frame no. 3. The marker no. 3 acts as a determinate point in frame no. 3. Role of the marker no. 5 is similar to marker no. 3. Displacements *d*_1_, *d*_3_, and *d*_4_ are calculated based on pixel locations of corresponding hinges.

By extracting edges corresponding to the upper boundary of links no. 0, 1, and 3, angle *θ*_1_ and sum *θ*_2_ + *θ*_3_ can be obtained. The orientation of frame no. 5 is determined by markers no. 4 and 5, since there is no straight upper boundary on link no. 5. The orientation of linear segment connecting those two markers is calculated based on markers' pixel location, then the sum *θ*_4_ + *θ*_5_ can be calculated.

Namely, all angular displacements can be directly extracted. When joints' angles are small, most parts of links no. 2 and 4 are obscured by adjacent links, the extraction precision would be low; therefore, special attention is paid to angles *θ*_2_ and *θ*_4_. Given equations (1)–(5), it is easy to obtain the following transformation matrices by matrices multiplication as:

(6) $$\begin{array}{c} T_{3}^{1}=\left[\begin{array}{ccc} c_{23} & -s_{23} & d_{1}+d_{2}\cos\theta_{2}+d_{3}c_{23}\\ s_{23} & c_{23} & d_{2}\sin\theta_{2}+d_{3}s_{23}\\ 0 & 0 & 1 \end{array}\right], \end{array}$$

(7) $$\begin{array}{c} T_{5}^{3}=\left[\begin{array}{ccc} c_{45} & -s_{45} & d_{4}+d_{5}\cos\theta_{4}\\ s_{45} & c_{45} & d_{5}\sin\theta_{4}\\ 0 & 0 & 1 \end{array}\right], \end{array}$$

where *c*_23_ and *s*_23_ are the abbreviations of terms cos(*θ*_2_ + *θ*_3_) and sin(*θ*_2_ + *θ*_3_), and other terms possess similar meaning.

Taking matrix *T*_3_^1^ as an instance, coordinates of a distinct point in frames no. 3 and 1 are denoted by *u*, *v*, *x*, and *y*, respectively (see Figure 5). The relationship between those quantities can be expressed as:

(8) $$\begin{array}{c} \left[\begin{array}{c} x\\ y \end{array}\right]=T_{3}^{1}∙\left[\begin{array}{c} u\\ v \end{array}\right]. \end{array}$$

More explicitly,

(9) $$\begin{array}{c} x=c_{23}u-s_{23}v+d_{1}+d_{2}\cos\theta_{2}+d_{3}c_{23}, \end{array}$$

(10) $$\begin{array}{c} y=-s_{23}u+c_{23}v+d_{2}\sin\theta_{2}+d_{3}s_{23}, \end{array}$$

where *u*, *v*, and *d*_2_ are known, variables *x*, *y*, *d*_1_, and *d*_3_ can be directly read from the image, the sum *θ*_2_ + *θ*_3_ also can be extracted with adequate accuracy, then *s*_23_ and *c*_23_ can be calculated. Finally, *θ*_2_ can be obtained as:

(11) $$\begin{array}{c} \theta_{2}=\arctan\left(\frac{y+s_{23}u-c_{23}v-d_{3}s_{23}}{x-c_{23}u+s_{23}v-d_{1}-d_{3}c_{23}}\right). \end{array}$$

Due to mechanical constraints, *θ*_2_ is valid only in the fourth quadrant, so there is a distinct solution of the function *arctan*() with only one argument.

Similarly, *θ*_4_ can be solved as:

(12) $$\begin{array}{c} \theta_{4}=\arctan\left(\frac{y+s_{45}u-c_{45}v}{x-c_{45}u+s_{45}v-d_{4}}\right), \end{array}$$

where *u* and *v* are constants defined in the fifth link coordinate frame, and *x* and *y* are expressed in the third link frame.

### 3.3. Data Fitting Function

Analytical expressions of variables should be obtained by fitting sample data. Based on preliminary experiments, piecewise polynomial functions are chosen. First, switching points are determined intuitively by observing the data curve, then, in each segment, the degree and corresponding parameters are obtained by the nonlinear least square method (LSM) [41]. For the same data set, a polynomial of degrees from 0 to 3 are implemented as the desired model, then the polynomial with the minimum squared error is adopted. This will be explained with examples in the next section.

## 4. Experimental Results

### 4.1. Experimental Setup

During the modeling process, the exoskeleton's palm is steadily fixed onto a test table, and the camera is supported by a tripod, so the relative pose between the camera and the exoskeleton palm is kept invariant. The motor's step length is 4 mm, so there are 20 samples for one-way inside a total motion range of 80 mm. Six sample images are shown in Figure 7.

Twenty-four healthy Asian volunteers are recruited, who are required to keep the forefinger relaxed to follow exoskeleton's movement. For each volunteer, complete motion series including forward and backward stages are executed three times. More information about volunteers is listed in Table 2.

It is quite easy to wear the glove because of a semiopen form for the finger part, that is, Velco is implemented to fasten (see Figure 6). For a healthy volunteer, it consumes less than 1 minute to wear with help of others.

### 4.2. Original Data and Fitting Functions

The curve of *d*_1_ of volunteer 1 during a forward movement is shown in Figure 8. The expression is consisted of three parts, with a form of constant, linear function and constant, respectively.

An interesting phenomenon is observed that for all configuration variables, there are obvious differences between forward and backward movements, either shift or shape deformation. To demonstrate this, the original data set and fitted curves for all eight configuration variables of volunteer 1 are drawn in Figures 9–10. Corresponding expressions are listed in Table 3, where the argument *x* represents the motor displacement. It is observed that for translational displacements *d*_1_, *d*_3_, and *d*_4_, differences are with the form of relative regular hysteresis. For angular variables, situation is more complicated. For *θ*_1_, shapes corresponding to two ways are totally different, so do the corresponding expressions. For *θ*_3_, expressions even possess different degrees.

Then, the repeatability for an individual volunteer is verified. As instances, *d*_1_ and *θ*_2_ of the volunteer 1 are shown in Figure 11. A similar phenomenon appears for other variables and volunteers. It can be seen that the repeatability is quite good, that is, data can be fitted by similar expressions.

Difference between volunteers is also analyzed. As an instance, the standard deviation of *d*_1_ and *θ*_5_ are shown in Figure 12. It can be found that the maximum for *d*_1_ takes place in the middle part, which is mainly caused by shift (see Figure 11(a)). And the standard deviation of *θ*_5_ increases with it. A similar phenomenon appears in rest variables. If necessary, the model for different volunteers can be described by the same type of expressions with different parameter values.

The relationship between the motor's displacement and the total flexing angle of the exoskeleton for volunteer 1 is shown in Figure 13. It can be observed that the nonlinearity is obviously weaker than relationships between motor displacement and most intermediate variables, and so does the difference between forward and backward movements. By LSM, the relationship can be described by:

(13) $$\begin{array}{c} \theta \left(x\right)=\left\{\begin{array}{c} -0.013x^{2}-1.05x-3.14,\;\;\text{forward}\\ -0.0083x^{2}-1.33x-8.52,\;\;\text{backward} \end{array}\right., \end{array}$$

where the total flexing angle is denoted by *θ*. Equation (13) can be employed as a kinematics model for rehabilitation trajectory generation or control purposes.

The standard deviation of *θ*(*x*) for all volunteers is shown in Figure 14. Similar to an individual angle, the standard deviation increased with *θ*(*x*), and the maximum reaches about 12 degrees, while the bending angle is nearly −160 degrees (see Figure 7). The ratio between standard deviation and the bending angle itself is shown in Figure 14(b). In the beginning, a big ratio is due to that the bending angle itself is small; therefore, the influence of noise is significant. With increasing *θ*(*x*), this ratio convergence to low level, that is, about 0.1. This phenomenon demonstrates that the exoskeleton possesses a good generality to volunteers. From a hardware point of view, it adapts to different finger lengths and length variations during movement. From a software point of view, it will be easy to “customize” a distinct finger model by calibration.

## 5. Conclusion

A robotic exoskeleton for fingers rehabilitation is introduced, which possesses the following characteristics:

- two links mimicking knuckles are implemented
- links are connected by passive joints
- bidirectional torque is exerted by one Bowden cable with help of a sleeve
- the maximum bending angle approaches nearly −160 degrees

Because of those characteristics, it possesses good adaptability to finger length of different subjects and length variation during movement while keeping the structure compact. Piecewise polynomial functions are chosen as the direct kinematics model. Experimental results show that this robot possesses adaptability to different subjects and has achieved nearly the maximum finger bending angle of a healthy adult person. It will be easy to customize a distinct finger model by calibration for the individual patient, individual finger, or during different therapy stages, to satisfy rehabilitation requirements.

## Figures and Tables

**Figure 1:** Mechanical structure of the finger rehabilitation exoskeleton.

**Figure 2:** Definition of links and coordinate frames for one finger.

**Figure 3:** Mechanical structure to guarantee cable stiffness.

**Figure 4:** Control system structure.

**Figure 5:** Definition of some kinematics variables.

**Figure 6:** A sample image of the robotic exoskeleton with five markers.

**Figure 7:** Images series acquired during the model building process.

**Figure 8:** Samples and the fitted curve of displacement *d*_1_ of volunteer 1.

**Figure 9:** Displacements measured in both forward and backward movements.

**Figure 10:** Angular displacements *θ*_*i*_ measured in both forward and backward movements.

**Figure 11:** Repeatability with respect to movement of volunteer no. 1.

**Figure 12:** Standard deviation of variables *d*_1_ and *θ*_5_ of all volunteers.

**Figure 13:** Finger's total flexing angle of volunteer 1.

**Figure 14:** Finger's total flexing angle of all volunteers.

**Table 1:** Geometrical parameters corresponding to the forefinger.

	Constant/variable	Value/range	Unit
*d*_1_	Variable	[18.5, 24.5]	mm
*d*_2_	Constant	30	mm
*d*_3_	Variable	[−4, 0.5]	mm
*d*_4_	Variable	[11.5, 16.0]	mm
*d*_5_	Constant	20	mm
*θ*_1_	Variable	[−20, 0]	Degree
*θ*_2_	Variable	[−20, 0]	Degree
*θ*_3_	Variable	[−60, 0]	Degree
*θ*_4_	Variable	[−30, 0]	Degree
*θ*_5_	Variable	[−50, 0]	Degree

**Table 2:** Some information with respect to volunteers.

	Gender		Age, years				Weight (kg)		
	Male	Female	18–30	31–40	41–50	>50	40–55	56–70	>70
Number	14	10	6	6	6	6	7	12	5
Percentage 5%	58%	42%	25%	25%	25%	25%	29%	50%	21%

**Table 3:** Expression of fitted joint variables.

	Forward	Backward
*d*_1_	$\left\{\begin{array}{c} 18.4\;\;\;\;\;0<\text{x}\leq 26\\ 0.27x+11.8\;26<x\leq 46\\ 24.6\;\;\;\;46<x<80 \end{array}\right.$	$\left\{\begin{array}{c} 18.4\;\;\;\;\;\;0<\text{x}\leq 8\\ 0.47x+15\;\;\;\;8<x\leq 18\\ 24.3\;\;\;\;\;\;18<x<80 \end{array}\right.$
*d*_3_	$\left\{\begin{array}{c} 0.2x-4.2\;\;0<x\leq 24\\ 0.6\;\;\;\;\;24<x<80 \end{array}\right.$	$\left\{\begin{array}{c} -4.1\;\;\;\;\;\;\;0<\text{x}\leq 16\\ 0.16x-6.5\;\;\;\;16<x\leq 44\\ 0.5\;\;\;\;\;\;\;44<x<80 \end{array}\right.$
*d*_4_	$\left\{\begin{array}{c} 0.0091x^{2}-0.12x+11.9\;0<x\leq 24\\ 15.7\;\;\;\;\;\;\;\;\;26<x<80 \end{array}\right.$	$\left\{\begin{array}{c} 11.5\;\;\;\;\;\;\;0<\text{x}\leq 26\\ 0.24x+5.4\;\;\;26<x\leq 42\\ 15.8\;\;\;\;\;\;42<x<80 \end{array}\right.$
*θ*_1_	−0.0019*x*^2^ − 0.056*x* − 0.82	$\left\{\begin{array}{c} -1.86\text{x}+2.4\;\;\;0<\text{x}\leq 6\\ -9.6\;\;\;\;\;\;6<x\leq 62\\ -0.446x+17.8\;\;62<x<80 \end{array}\right.$
*θ*_2_	−0.0001*x*^3^ + 0.01*x*^2^ − 0.47*x* − 0.4	−0.0001*x*^3^ + 0.013*x*^2^ − 0.72*x* − 3.1
*θ*_3_	−0.0082*x*^2^ − 0.12*x* − 0.6	−0.0002*x*^3^ + 0.02*x*^2^ − 1.05*x* + 4.5
*θ*_4_	$\left\{\begin{array}{c} 2.0\;\;\;\;\;\;\;0<\text{x}\leq 40\\ -0.97x+42.5\;\;\;40<x\leq 64\\ -23.8\;\;\;\;\;\;64<x<80 \end{array}\right.$	$\left\{\begin{array}{c} -2.3\;\;\;\;\;\;\;0<\text{x}\leq 34\\ -0.77x+25.6\;\;\;34<x\leq 62\\ -23.9\;\;\;\;\;\;62<x<80 \end{array}\right.$
*θ*_5_	0.0044*x*^2^ − 0.91*x* − 0.1	−0.0021*x*^2^ − 0.49*x* + 1.5

## Data Availability

The data used to support the findings of this study are available from the corresponding author.
